# Intervention Study of Dictyophora Polysaccharides on Arsenic-Induced Liver Fibrosis in SD Rats

This article has been retracted.

**DOI:** 10.1155/2022/7509620

**Published:** 2022-03-30

**Authors:** Guoze Wang, Peipei Zuo, Kai Ding, Qibing Zeng, Ting Hu, Shaofeng Wei, Peng Luo

**Affiliations:** ^1^The Key Laboratory of Environmental Pollution Monitoring and Disease Control, Ministry of Education & Affiliated Hospital of Guizhou Medical University & School of Public Health, Guizhou Medical University, Guiyang 550025, China; ^2^State Key Laboratory of Functions and Applications of Medicinal Plants, Guizhou Medical University, Guiyang 550014, China; ^3^Guizhou Provincial Engineering Research Center of Food Nutrition and Health, Guiyang, 550025 Guizhou, China

## Abstract

Long-term arsenic (As) exposure can cause liver injury, hepatic cirrhosis, and cancer. Meanwhile, Dictyophora polysaccharides (DIP) have excellent antioxidation, anti-inflammation, and immune protection effects. There are currently few reports on the protection effects of DIP on As-induced hepatotoxicity and its pharmacological value. Therefore, this study was aimed at elucidating the protection of DIP on As-induced hepatotoxicity and exploring its preventive role in antifibrosis. In our study, the SD rat As poisoning model was established by the feeding method to explore the influence of As exposure on liver fibrosis. Then, DIP treatment was applied to the rats with As-induced liver fibrosis, and the changes of serum biochemical indexes and liver tissue pathology were observed. And the expression of fibrosis-related proteins TGF-*β*1, CTGF, and *α*-SMA levels was then determined to explore the DIP intervention function. The results demonstrated that through reduced pathological changes of hepatic and increased serum AST, ALT, TP, ALB, and A/G levels, DIP ameliorated liver fibrosis induced by As as reflected. And the administration of DIP decreased the concentration of HA, LN, PCIII, CIV, TBIL, and DBIL. In addition, the synthesis of TGF-*β*1 inhibited by DIP might regulate the expression of CTGF and decrease the proliferation of fibrinogen and fibroblasts, which reduced the synthesis of fibroblasts to transform into myofibroblasts. And a decrease of myofibroblasts downregulated the expression of *α*-SMA, which affected the synthesis and precipitation of ECM and alleviated the liver fibrosis caused by exposure to As. In conclusion, based on the pathological changes of liver tissue, serum biochemical indexes, and related protein expression, DIP can improve the As-induced liver fibrosis in rats and has strong medicinal value.

## 1. Introduction

Arsenic (As) is a metallic element widely found in the natural environment, including the earth's crust, soil, groundwater, ambient air, and living organisms [1]. The different forms of As can migrate and accumulate in the atmosphere, soil, and water. Generally, As has different physical and chemical factors that result in various degrees of environmental toxicity [2]. The primary sources of As include natural sources and artificial sources (industrial and agricultural release). With the rapid development of modern agriculture and industry, arsenide compounds are widely used in nonferrous metals, pigments, fuels, glass, and pesticides. However, they cause various environmental pollutions, including air, soil, groundwater, and food [3]. As is a serious threat to human health; therefore, studies have increasingly focused on how to treat and prevent As poisoning.

Long-term exposure to As or arsenide compounds and consumption of As-exposed food cause severe harm to humans and animals, including diabetes, neurological diseases, various forms of cancer, cardiovascular diseases, and peripheral vascular diseases [4, 5]. Previous epidemiological investigations and animal experiments have confirmed that As is correlated with liver damage. Research has shown that the occurrence and development of liver diseases caused by acute and chronic As poisoning are associated with the synthesis and metabolism of cytokine regulatory networks composed of many proinflammatory and anti-inflammatory cytokines [6]. Meanwhile, As and its metabolites are toxic to hepatocytes, cause DNA damage, and produce several free radicals. The free radicals subsequently induce lipid peroxidation, which can cause cell dysfunction or directly attack the cells, triggering their damage [7]. Hepatocytes are repeatedly damaged and repaired, resulting in hepatic fibrosis [8]. Some studies also found that liver fibrosis is a reversible pathological process, and it is necessary that hepatic stellate cells reverse to their static state during liver fibrosis [9]. At present, research on As and arsenide compounds poisoning is limited.

Recently, numerous studies have confirmed that chronic As poisoning could induce liver injury. The effect of “As expulsion therapy” in managing chronic As poisoning is effective but has certain limitations. Research has established that the pectic polysaccharides of Momordica charantia could inhibit the oxidative stress of liver cells induced by sodium arsenite [10]. Besides, numerous studies have demonstrated that polysaccharides regulate immunity and protect the liver [11, 12]. Hence, our study explored effective and side effect-free hepatoprotective regimens from natural active products to manage chronic As poisoning.

Dictyophora is a cryptophytic root-parasitic fungus on withered bamboo. In Guizhou Province, five different types of Dictyophora are edible and medicinal. Dictyophora is rich in nutrition and fragrance and has a delicious taste. Generally, it is known as “flower of fungi” or “queen of fungi” [13]. In addition, some research has shown that Dictyophora is rich in amino acids, vitamins, polysaccharides, and inorganic salts. The dried Dictyophora contains protein, fat, total carbohydrate, bacterial sugar, crude fiber, and ash at concentrations of 19.4%, 2.6%, 60.4%, 4.2%, 8.4%, and 9.3%, respectively [14]. Among them, polysaccharide is a polyhydroxy aldehyde ketone polymer formed by ten or more monosaccharides through glycosidic bonds. It widely exists in higher plants, animal cell membranes, and microbial cell walls [15]. Furthermore, polysaccharides have many biological activities such as antioxidation, enhancing immunity, antitumor, neuroprotection, and antiaging [16]. In particular, studies have discovered that DIP have positive effects on liver damage [17]. The results of animal experiment in vivo showed that treatment with DIP could improve the excessive level of lipid profiles in liver injury caused by hyperlipidemia, as well as strengthen antioxidant status [18]. Meanwhile, DIP administration could improve obesity-associated hepatic metabolic impairment and ameliorate oxidative stress of liver by downregulating serum enzyme activities [19]. At present, many scientists have turned their attention to fungus polysaccharides, because they are natural and free of harmful side effects and have highly effective antioxidant properties. Moreover, their extraction process is relatively simple with minimal toxicity and side effects.

This study used rats whose metabolism mimics that of humans to comprehensively evaluate the relative efficacy function of DIP on As-induced liver injury. It has used the feeding method to establish an As poisoning model, which explores the influence of As on liver damage and evaluates the degree of liver fibrosis. Subsequently, after the intervention of DIP, we observed changes in serum biochemical indexes and pathological liver tissues. Taken together, our research has established that DIP have functional protective effects on As-induced liver injury in rats, and this function may regulate the expression of fibrosis-related proteins. Furthermore, this is the first study to explore the efficacy of different DIP levels on As-induced liver injury, providing new natural drug treatment insights for chronic As poisoning. Lastly, it gives a theoretical basis to advance the medicinal value of DIP.

## 2. Materials and Methods

### 2.1. Ethics Statement

This study was approved by the Guizhou Medical University experimental animal operation regulations and welfare management committee. All methods used herein were performed in accordance with the relevant guidelines.

### 2.2. Animal Grouping and Treatment

The study rats were randomly allocated into four groups and exposed to sodium arsenite (Sigma, USA, serial number: C1386-50G, purity: 98.9%) by feeding for three months at doses of 0, 25, 50, and 100 mg/kg. Subsequently, forty SD rats in the medium As group were randomly divided into four groups (*n* = 10 in each group, half male and half female) and exposed to DIP. Water extraction and alcohol precipitation methods were applied to extract DIP from Dictyophora, and the extraction rate was 13.016%. The detailed extraction steps and structure of DIP were reported in previous research by our research group [20]. DIP administration was by gavage once a day for 30 d, at a dose of 0, 2.5, 5, and 10 mg/ml (20 ml/kg BW). All rats were fed with a normal diet and free water.

### 2.3. Organization of Sample Collection

The experiment endpoint was fasting rats for 12 h, after which the weight of each group was measured. Cardiac blood was collected by an EDTA tube, centrifuged at 3000 rpm for 10 min, and stored at -80°C. After the rats were killed, the livers were separated, and the livers in each group were weighed. The liver weight of each group was calculated as liver weight/rat weight, using the unit grams per 100 g BW.

### 2.4. Analysis of Total As Content

The As content in the sample was determined by incomplete digestion flame atomic absorption spectrometry (AF-630A, Beijing Rayleigh Analytical Instrument Co, Ltd, China). Firstly, the 200 mg liver tissue was put in a clean 2 ml EP tube and ground with an electronic homogenizer. Then, a 7 ml nitric acid solution was added, and the tissue was fully digested in a microwave digester for 3 h. The samples were then stored for further determination.

### 2.5. Serum Biochemistry

The blood samples were collected from the cardiac apex, and plasma samples were obtained by centrifugation at 3000 rpm for 10 min, then used to obtain serum samples. The serum was used for measurement of alanine aminotransferase (ALT), aspartate aminotransferase (AST), total protein (TP), albumin (ALB), total bilirubin (TBIL), and direct bilirubin (DBIL) by an automatic biochemical analyzer (AU400, Olympus Co, Ltd, Japan). Subsequently, four indexes of serum liver fibrosis, including hyaluronic acid (HA), laminin (LN), type III collagen (PC), and type IV collagen (CIV), were detected by ELISA Kits (Wuhan bode Bioengineering Co, Ltd, China).

### 2.6. H&E and Masson Staining

For each experimental group, a small piece of liver tissue was sampled from the left liver lobe and fixed in 4% formalin. After 24 h, the tissues were dehydrated in 70%, 80%, 90%, 95%, and 100% ethanol series and embedded in paraffin; then, 5-micron serial sections were sliced on a microtome. The sections were in turn dehydrated by graded ethanol (95%, 75%, 45%, and 25%), vitrificated by dimethylbenzene and wax immersion, and subjected to routine HE staining. After dehydration in ethyl alcohol, the sections were stained with a nuclear dye solution for 2 min, followed by cytoplasmic dye for 1 min. Afterward, the sections were stained with color separation solution and redyeing solution for 5 min at room temperature. The sections were then observed under a light microscope (BX51, Olympus, Japan, 400x). Histopathological scores were calculated with reference to Additional Table 1 and Additional Table 2.

### 2.7. Immunohistochemistry Analyses of TGF-*β*1, CTGF, and *α*-SMA

Immunohistochemistry staining was performed using the previously prepared paraffin sections. The stained sections were observed under the light microscope (BX51, Olympus, Japan, 400x). The integrated optical density (IOD) and area of all the collected images were measured by an Image-Pro Plus 6.0 image analysis system.

### 2.8. Statistical Analysis

The data are presented as the mean ± SEM. The comparisons among several groups were performed by one-way ANOVA using SPSS 17.0. Pairwise comparison and analysis of homogeneous variance were conducted using LSD, while uneven variance was analyzed by the Games-Howell method. *P* < 0.05 was considered statistically significant.

## 3. Results

### 3.1. Basic Information of Rats

All 80 SD rats survived. Compared with the control group, the low and medium As groups demonstrated slower weight gain, had medium body shape, and slightly sparse hair. Meanwhile, the high As group had very slow growth, extremely dim and sparse hair, and obvious depilation on the back and buttocks. The high As group rats demonstrated poor spirit, normal walking, and reduced activity. With time increment, the food intake of the control group increased significantly (*P* < 0.05). However, the food intake of rats in the high As group showed a significant (*P* < 0.05) downward trend with the increase of exposure dose and time (Figures 1(a) and 1(b)). Weekly evaluation of the rodent weights in the As poisoning group showed a slow increase with the increase of dose and time (Figures 1(c)).

### 3.2. DIP Ameliorates Liver Coefficient and As Content by As-Induced Liver Injury in Rats

This study evaluated the liver coefficient and As contents to assess the protective effects of DIP against As-induced injury in rats. As shown in Figure 2(a), the liver coefficient increased significantly with an increase in the As exposure dose (*P* < 0.05). Furthermore, the As content in the liver also increased significantly with an increase of exposure dose, relative to the control group (*P* < 0.05) (Figure 2(b)). Intervention with DIP resulted in a significant decrease (*P* < 0.05) of the liver coefficient of the treatment group (Figure 2(c)); the change was more substantial with increase in the polysaccharide dose. Meanwhile, the As content decreased with increase in the DIP concentration; there were significant differences between the As high-dose group and its control group (*P* < 0.05) (Figure 2(d)).

### 3.3. DIP Ameliorates As-Induced Liver Injury in Rats

In order to investigate the protective effect of DIP in As-induced liver injury, we assessed the liver histopathological changes; the serum ALT, AST, TP, A/G, and ALB; and bilirubin metabolism levels of TBIL and DBIL. Histological analysis by H&E staining in the low As group showed an increase in the volume of hepatocytes; the cytoplasm stained lightly and loosely than the control group (Figures 3(a)–3(d)). Meanwhile, hepatic edema and vacuolar degeneration could be observed. The results of the medium As group suggested that the volume of hepatocytes expanded further due to hepatocyte hydrodenaturation. Also, the hepatocytes showed varying degrees of edema and vacuolar degeneration and inflammatory cell infiltration in the stroma; hepatocyte liquefaction and necrosis were apparent. The results showed that hemangiectasis was more obvious in the high As group than in the medium-dose group. Besides, cell swelling, inflammatory cell infiltration, fiber hyperplasia, and other unique cell trauma characteristics were more apparent in the high As group. The As groups demonstrated a dose-dependent remarkable increase in the levels of serum ALT and AST (*P* < 0.05) (Figure 4(a)) and the bilirubin metabolism of TBIL and DBIL (*P* > 0.05) (Figures 4(c)); however, the TP, A/G, and ALB levels of As groups decreased to varying degrees, relative to the control (*P* < 0.05) (Figure 4(e)). Administering DIP significantly diminished the levels of ALT, AST, TBIL, and DBIL and increased the levels of TP, A/G, and ALB in the serum (*P* < 0.05) (Figures 4(b), 4(d), and 4(f)). Increasing the DIP dose decreased the collagen fibers around the hepatic lobule and the portal area, and inflammatory cell infiltration also decreased (Figures 3(e)–3(g)). These results suggest that DIP plays a protective role in mitigating As-induced liver injury in rats.

### 3.4. DIP Ameliorates As-Induced Liver Fibrosis in Rats

We detected four markers of liver fibrosis in serum to further evaluate the degree of liver fibrosis in rats. The results showed that the concentrations of LN, HA, PCIII, and CIV had a significant increasing trend relative to the control group (*P* < 0.05) (Figure 5(a)). We also performed Masson staining to precisely confirm the results of liver fibrosis. In turn, we observed a few blue-stained collagen fibers around the hepatic lobule and portal area, and the collagen fibers around the hepatic lobule were slightly proliferated in the low As group (Figure 6(b)). The results of the medium As group revealed significant inflammatory cell infiltration in the interstitium, with moderate hyperplasia of collagen fibers around liver lobules (Figure 6(c)). Moreover, a large number of fibrous septa formed in the peripheral area of the lobules, and there was obvious inflammatory cell infiltration in the interstitium of the high As group. Meanwhile, the collagen fibers around the hepatic lobules were moderately and severely proliferated (Figure 6(d)). According to the image analysis system, the area of proliferative fiber in the liver of rats increased with increasing exposure dose. There were statistically significant differences in the area of collagen fiber deposition in the low, medium, and high As groups, compared with the control group (*P* < 0.05) (Figure 6(h)). In brief, degeneration and liver fibrosis demonstrated an inevitable surge with increasing concentration of sodium arsenite. DIP treatment reversed the levels of LN, HA, PCIII, and CIV caused by chronic As exposure (Figures 5(b)). Subsequently, fibrous tissue hyperplasia of hepatocytes in the treatment group was significantly less than that in the As poisoning group (Figures 6(e)–6(g)). Meanwhile, the area of proliferative fiber in the liver of rats decreased after the administration of DIP; there were statistically significant differences among the low-, medium-, and high-dose polysaccharide groups relative to the As poisoning control group (*P* < 0.05) (Figure 6(i)).

### 3.5. DIP Inhibits the Expression of Fibrosis-Related Protein TGF-*β*1, CTGF, and *α*-SMA Levels

To further determine the antifibrosis function of DIP-triggered inhibition of TGF-*β*1, CTGF, and *α*-SMA expression, we evaluated the expression levels of these proteins in rat livers. TGF-*β*1 was only slightly expressed in the portal area and the wall of the central lobular vein in the control group; however, its expression increased with an increase in the As dose. The TGF-*β*1-positive cells were mostly concentrated in the portal area and proliferative collagen fibers, with a clear contour **(**Figures 7(a)–7(d)). The optical densities of TGF-*β*1 proteins from the livers of As-treated rats were significantly higher than those from control livers (*P* < 0.05) (Table 1). In addition, CTGF was expressed in liver parenchymal cells and stromal cells of the portal area, as demonstrated by a brownish-yellow coloration in positive regions. The expression of CTGF increased with increase in the exposure dose, and the positive cells were mostly concentrated in the interstitial cells of the portal area, with a clear contour (Figures 8(a)–8(d)). We also found that the optical density of CTGF protein expression increased significantly (*P* < 0.05) with increase in exposure dose (Table 1). *α*-SMA was expressed in the cell membrane or cytoplasm, and its positive products were yellow and brown. In the medium and high As groups, *α*-SMA had high expression in the cell membrane and cytoplasm. The expression of *α*-SMA showed an increased response in a dose-dependent manner according to the As concentration (Figures 9(a)–9(d)). The optical density of the *α*-SMA protein was also significantly higher than that of the control group (*P* < 0.05) (Table 1). However, DIP posttreatment decreased the expression of TGF-*β*1, CTGF, and *α*-SMA proteins in the liver of rats, and the optical densities showed statistically significant decrease with increase in the DIP dose (*P* < 0.05) (Figures 7–9(e)–9(g), Table 2). These data indicate that DIP intervention could inhibit the expression of TGF-*β*1, CTGF, and *α*-SMA proteins, combined with the results of four indicators of fibrosis LN, HA, PCIII, and CIV concentration; DIP has the function of antifibrosis and liver protection.

## 4. Discussion

The liver is one of the main detoxification organs in the human body. In long-term chronic As poisoning, substantial amounts of organic As can be oxidized (III)As to (V)As by metabolizing the liver and reduced (V)As to (III)As or As methylation [21, 22]. Dictyophora contains a variety of trace elements and nutrients. And its polysaccharide is a high bioactivity macromolecule with high curative effects in lowering blood pressure, blood sugar, antitumor, and immune stimulation [23]. Our previous studies have shown that DIP intervention on As-induced L-02 cells alleviates the changes in cell viability, apoptosis, and oxidation stress [24]. Meanwhile, DIP could reduce arsenic content in the liver, increase As in blood and urine, and inhibit liver tissue damage caused by sodium arsenite [25, 26], suggesting that DIP could inhibit As toxicity at cellular and whole-organism levels and protect liver function. Therefore, on the basis of the previous, we explored the DIP that had a substantial protective effect on the occurrence and development of As-induced liver fibrosis in the present study.

We established a rat model of As poisoning by the feeding method, the research results showed that As contents and organ coefficient of the liver increase in each As-exposed group of rats, and the trend of weight gained slowly. The serum hepatic enzyme indexes of ALT and AST and metabolic levels of TBIL and DBIL in bilirubin increased, while the TP, A/G, and ALB levels decreased at varying degrees. These results indicated that the rats in each exposure group had different degrees of liver damage. (III)As exposure significantly increased the levels of serum biochemical indexes, which is consistent with previous study findings [27]. The DIP was entered intervention treatment after three months. Compared with the As poisoning control group, the protective effect on the liver injury was more obvious with increasing dose of DIP, suggesting that DIP has antagonistic effects on As-induced liver injury in rats.

Liver fibrosis refers to the pathological process of inflammation and necrosis of hepatocytes caused by various factors, which lead to the deposition of extracellular matrix (ECM), cytokine imbalance, and generation of liver fibroblasts [28]. Hence, liver fibrosis induced by sodium arsenite is a slow disease process in which many cellular and inflammatory factors participate, including hepatocyte hydrodegeneration, hepatocyte ballooning, hepatocyte necrosis (inflammatory infiltration), hepatocyte regeneration, fibrous tissue proliferation, and liver fibrosis [29]. There are four serum indicators for liver fibrosis, LN, HA, PCIII, and CIV. HA is a matrix component synthesized by stromal cells; it can accurately and sensitively reflect the amount of fiber produced in the liver and the damage extent of liver cells, which is a sensitive index of liver fibrosis and cirrhosis [30]. CIV is the standard of collagen synthesis and the primary component of basement membrane reticular structure. In the initial stage of liver fibrosis, CIV proliferates and transforms rapidly and finally forms an extensive basement membrane with the precipitation of LN [31]. In this study, the concentrations of LN, HA, PCIII, and CIV in As-exposed groups increased with increase in the exposure dose; there was a positive correlation. This finding suggests that long-term As exposure can induce hepatic fibrosis. These findings are consistent with Tao et al.'s results that long-term exposure to sodium arsenite can induce hepatic stellate cell (HSC) activation and hepatic fibrosis in SD rats [32]. Combined HE and Masson staining can accurately determine the level of tissue fibrosis. The current study showed that liver fibrosis aggravates the degeneration and necrosis of liver cells and inflammatory cell infiltration with prolonged As exposure time. A large number of fibrous septa and moderately to severely proliferated collagen fibers formed around the hepatic lobules. Meanwhile, the structure of liver lobules was abnormal, and the cell lines had a disordered arrangement. It is obvious that inflammatory cells infiltrate the interstitial tissues, accompanied by a progressive increase of fibrous tissue proliferation. This result suggested that As exposure could cause liver injury in rats, and the degree of liver fibrosis was aggravated with increase in dose and time. Intervention with DIP decreased the concentrations of LN, HA, PCIII, and CIV with increasing polysaccharide doses. Following intervention, the collagen fibers in the peripheral and portal areas of the liver lobule and inflammatory cells decreased, and the area of hyperplastic fiber demonstrated a reducing trend, suggesting that DIP has antagonistic effects on the progression of liver fibrosis.

When the damage of inflammatory cells and damage factors (alcohol, virus, drugs, poisons, parasites, etc.) to the liver exceeds the compensatory capacity of the body, it releases various inflammatory factors, activating HSC to transform into myofibroblast cells, further leading to substantial precipitation of ECM and proliferation of fibrous connective tissue. And the reconstructed hepatic lobules and formed pseudolobules or nodules develop into liver fibrosis, cirrhosis, and liver cancer, eventually leading to liver failure and death. However, synthesis and degradation of ECM are mainly controlled by TGF-*β*1. When liver injury occurs, activation of hepatocyte leads to the increase of TGF-*β*1 synthesis, with aggravating degree of fibrosis; CTGF was found to be overproduced in liver tissue. CTGF is an important downstream factor that mediates the profibrotic effect of TGF-*β*1 and regulates the growth of fibroblasts and the secretion of ECM. Both TGF-*β*1 and CTGF can stimulate the synthesis of fibroblasts to transform into myofibroblasts, thus upregulating the expression of *α*-SMA and increasing the synthesis of ECM [33, 34] (Figure 10). As an important fibrosis cytokine, TGF-*β*1 is an initiating factor of liver fibrosis [35]. The protein expression was located in the cell cytoplasm, and the positive products were brown-yellow. Since TGF-*β*1 plasma concentrations can be significantly increased and are closely related to ALT and AST levels in severe liver injury, the protein TGF-*β*1 is a marker of liver inflammation and necrosis [36]. Our results showed that the expression of TGF-*β*1 increased with increasing exposure dose in the liver tissue of rats. The TGF-*β*1-positive cells were mostly concentrated in the portal area and proliferative collagen fibers with a clear outline. CTGF is a strong, sensitive index for expression, mainly expressed in the liver parenchymal cells and interstitial cells in the portal area. The CTGF-positive product is brown-yellow, while strongly positive is brown. We found high expression in the portal area and cytoplasm in the moderate and high As-exposed group, and the positive cells were mainly concentrated in the interstitial cells. The expression of *α*-SMA was located in the cell membrane or cytoplasm; its positive products are yellow and brown. We found high *α*-SMA expression in the membrane and cytoplasm of medium and high As-exposed groups. The expression level of *α*-SMA in the liver of rats increased with increasing exposure dose. DIP intervention decreased the expression of TGF-*β*1, CTGF, and *α*-SMA protein in rat liver. The combined results of the four serum liver fibrosis indexes, LN, HA, PCIII, and CIV, suggested the synthesis of TGF-*β*1 inhibited by DIP might regulate the expression of CTGF and decrease the proliferation of fibrinogen and fibroblasts, which reduced the synthesis of fibroblasts to transform into myofibroblasts. And a decrease of myofibroblasts downregulated the expression of *α*-SMA, which affected the synthesis and precipitation of ECM and alleviated the liver fibrosis caused by exposure to As. The activation of cytokines may relate to the regulation of relevant pathways, which needs further study.

Taken together, long-term exposure of SD rats to sodium arsenite by the feeding method can cause liver damage, and the degree of harmful effects is positively correlated with the concentration of As. The current study results demonstrated that DIP mitigated the serum AST, ALT, TP, ALB, A/G, TBIL, and DBIL levels and the concentrations of HA, LN, PCIII, and CIV. Thus, DIP alleviates the liver histopathological changes caused by exposure to As. Further study indicated that DIP significantly inhibited As-induced liver fibrosis by decreasing the expressions of fibrosis-related proteins TGF-*β*1, CTGF, and *α*-SMA. This finding suggests that DIP could regulate the synthesis and degradation of ECM and inhibit fibroblast proliferation, which alleviated the liver fibrosis caused by exposure to As. Combined with the results of our previous research, the current study findings suggest that DIP has excellent prospects for application in protecting the liver.

## Figures and Tables

**Figure 1:** General situation of rats by sodium arsenic: (a) As group rats of changes in food intake; (b) As group rats of average daily taken As content; (c) As group rats of weight trend chart. Values are mean ± standard deviation, and *n* = 10. ^∗^*P* < 0.05.

**Figure 2:** Organ coefficient and As content in liver of rats: (a, b) changes of the rat liver coefficient and the As content in the liver in the model group; (c, d) changes of the rat liver coefficient and the As content in the liver in the DIP group. Values were mean ± standard deviation, and *n* = 10. ^∗^*P* < 0.05.

**Figure 3:** HE staining of the liver: (a) the control group; (b) the low As group; (c) the medium As group; (d) the high As group; (e) the low DIP group; (f) the medium DIP group; (g) the high DIP group (HE ×100).

**Figure 4:** Serum-related indexes of liver injury in rats: (a) changes of the rat liver damage index of serum enzymology in the model group; (b) changes of the rat liver damage index of serum enzymology in the DIP group; (c) changes of bilirubin metabolism in the model group; (d) changes of bilirubin metabolism in the DIP group; (e) changes of protein synthesis function in the model group; (f) changes of protein synthesis function in the DIP group. Values are mean ± standard deviation, and *n* = 10. ^∗^*P* < 0.05.

**Figure 5:** Changes of four indexes of liver fibrosis in rats. (a) Changes of four indexes of liver fibrosis in the model group. (b) Changes of four indexes of liver fibrosis in the DIP group. Values are mean ± standard deviation, and *n* = 10. ^∗^*P* < 0.05.

**Figure 6:** Masson staining of the liver: (a) the control group; (b) the low As group; (c) the medium As group; (d) the high As group; (e) the low DIP group; (f) the medium DIP group; (g) the high DIP group (Masson ×100); (h) the rat liver hyperplasia of fibrous tissue area measurement in the model group; (i) the rat liver hyperplasia of fibrous tissue area measurement in the DIP intervention group. Values are mean ± standard deviation, and *n* = 10. ^∗^*P* < 0.05.

**Figure 7:** Immunohistochemical staining of TGF-*β*1: (a) the control group; (b) the low As group; (c) the medium As group; (d) the high As group; (e) the low DIP group; (f) the medium DIP group; (g) the high DIP group (×400).

**Figure 8:** Immunohistochemical staining of CTGF: (a) the control group; (b) the low As group; (c) the medium As group; (d) the high As group; (e) the low DIP group; (f) the medium DIP group; (g) the high DIP group (×400).

**Figure 9:** Immunohistochemical staining of *α*-SMA: (a) the control group; (b) the low As group; (c) the medium As group; (d) the high As group; (e) the low DIP group; (f) the medium DIP group; (g) the high DIP group (×400).

**Figure 10:** Schematic diagram of hepatic fibrosis-related proteins. The inflammatory cells and damage factors can activate HSC in liver tissue and increase the synthesis of TGF-*β*1, which led to proliferation of fibrous connective tissue and upregulated the expression of CTGF. And the synthesis and transformation of fibroblasts into myofibroblasts, thereby regulating the expression of *α*-SMA, were increased the synthesis of ECM and caused liver fibrosis finally.

**Table 1:** TGF-*β*1-, CTGF-, and *α*-SMA-positive color intensity and density value in the As model group (*n* = 10, $\bar{x}\pm s$).

Group	TGF-*β*1		CTGF		*α*-SMA	
	Immune intensity	Density value	Immune intensity	Density value	Immune intensity	Density value
Control	+	150.45 ± 3.14	+	118.48 ± 9.52	+	123.63 ± 7.42
The low AS group	+~++	157.23 ± 2.29^a^	+~++	135.23 ± 10.13^a^	+	130.56 ± 9.15
The medium AS group	+~++	160.67 ± 1.24^a^	++~+++	156.47 ± 11.24^a^	+~++	155.85 ± 8.84^a^
The high AS group	++~+++	166.76 ± 3.34^a^	++~+++	164.25 ± 9.34^a^	+~+++	168.25 ± 11.34^a^

Note: ^a^compared with the normal group, *P* < 0.05. ^b^Compared with the As control group, *P* < 0.05.

**Table 2:** TGF-*β*1-, CTGF-, and *α*-SMA-positive color intensity and density value in the DIP group (*n* = 10, $\bar{x}\pm s$).

Group	TGF-*β*1		CTGF		*α*-SMA	
	Immune intensity	Density value	Immune intensity	Density value	Immune intensity	Density value
Control	+	149.34 ± 2.42	+	110.07 ± 11.02	—	131.19 ± 10.57
AS control group	+~+++	161.49 ± 1.13^a^	++~+++	149.34 ± 10.13^a^	++	159.36 ± 11.13^a^
The low DIP group	+~+++	158.67 ± 1.07	+~+++	141.22 ± 13.82	+~++	155.03 ± 9.88
The medium DIP group	+~++	154.44 ± 2.24^b^	+~++	132.29 ± 10.24^b^	+~++	137.55 ± 10.24^b^
The high DIP group	+~++	151.82 ± 2.82^b^	+~++	128.01 ± 11.34^b^	+	127.25 ± 12.18^b^

Note: ^a^compared with the normal group, *P* < 0.05. ^b^Compared with the As control group, *P* < 0.05.

## Data Availability

The data presented in this study are available on request from the corresponding author.

## Supplementary Materials

Supplementary Materials Supplementary 1. Supplementary Table 1: the histopathological scoring system in the As model group. Supplementary 2. Supplementary Table 2: the histopathological scoring system in DIP intervention.
